# Mucinous tubular and spindle cell renal cell carcinoma: a review of clinicopathologic aspects

**DOI:** 10.1186/s13000-015-0402-1

**Published:** 2015-09-17

**Authors:** Ming Zhao, Xiang-lei He, Xiao-dong Teng

**Affiliations:** Depatment of Pathology, Zhejiang Provincial People’s Hospital, Hangzhou, 310014 China; Department of Pathology, The First Affiliated Hospital, Zhejiang University College of Medicine, Hangzhou, 310003 China

## Abstract

Mucinous tubular and spindle cell renal cell carcinoma is a rare, recently described variant of renal cell carcinoma characterized by an admixture of cuboidal cells in tubules and sheets of spindle cells, and variable amounts of mucinous stroma. It has been recognized as a distinct entity in the 2004 World Health Organization tumor classification. Since then, several dozen of these tumor have been reported with additional complementary morphologic characteristics, immunohistochemical profile, and molecular genetic features that have further clarified its clinicopathologic aspects. Although originally considered as a low grade renal cell carcinoma on the basis of its bland appearing nuclear features and indolent clinical course, mucinous tubular and spindle cell renal cell carcinoma has currently been proven to be a tumor that has a histological spectrum ranging from low to high grade that includes sarcomatoid differentiation. In this review, we present a detailed summary of the current knowledge regarding the clinicopathologic, immunohistochemical, molecular genetic, and prognostic characteristics, as well as differential diagnoses of mucinous tubular and spindle cell renal cell carcinoma.

## Introduction

Mucinous tubular and spindle cell renal cell carcinoma (MTSRCC) is a rare and recently described subtype of renal cell carcinoma (RCC), which is recognized as a distinct entity in the 2004 *World Health Organization* (WHO) tumor classification [1]. As its descriptive namesake has indicated, this tumor is morphologically composed of three salient elements: tubules, spindle cells and extracellular mucinous/myxoid stroma. Previously, tumors showing a similar morphology had been referred to under a variety of rubrics including low-grade collecting duct carcinoma [2], low-grade myxoid renal epithelial neoplasm with distal nephron differentiation [3], low-grade tubular mucinous renal neoplasm and spindle and cuboidal renal cell carcinoma [4, 5]. To date, less than 100 cases of these tumor have been reported in the English language literature. In this review, we present a detailed summary of the current knowledge regarding the clinicopathologic, immunohistochemical, molecular genetic, and prognostic characteristics, as well as differential diagnoses of MTSRCC.

## Review

### Clinical characteristics

MTSRCC predominantly affects adult patients with a wide age range from 13 to 82 years (mean 53) and shows a female predominance with a 1:4 male-to-female ratio [6–8]. Although some tumors are symptomatic, such as flank pain, abdominal mass and hematuria [3], the majority are discovered incidentally during abdominal imaging studies for other unrelated reasons [9]. An association with nephrolithiasis [5] and those arising from the background of end stage renal disease have been noted [10]. Radiologically, MTSRCC displays a common appearance that is different from clear-cell RCC but similar to papillary RCC [11]. It usually presents as a well-demarcated, exophytic or partially exophytic renal mass and showes an expansile growth pattern with a spherical or ovoid shape on computed tomograph scan. Tumors less than 5-cm usually demonstrate homogenous pattern of enhancement while those larger than 5-cm often show heterogeneous enhancement pattern [11].

### Pathological findings

Grossly, the epicenter of MTSRCC is usually located in renal cortex. The tumors are generally well circumscribed and partially encapsulated, with a wide size range from less than 1-cm diameter to greater than 18-cm. The cut surface is commonly bulging, shiny and mucoid, with a uniform homogenous tan, gray or pale yellow color and a solid consistency [7, 9, 8, 12] (Fig. 1). Foci of hemorrhage and/or necrosis may be seen, but these are uncommon [7].

**Fig. 1:** Gross appearance of MTSRCC. The tumor is usually well-demarcated with a homogeneous, gray to white, often bulging and shiny mucoid cut surface

Histologically, the tumor is characterized by a mixture of tubular and spindle cell components separated by variable amounts of mucinous stroma [12, 7, 8] (Fig. 2). The tubules are round, ovoid, or elongated with a collapsed central lumen, they are usually tightly packed and parallelly arranged, and sometimes merge into cord-like structures or even form a solid growth pattern (Fig. 2a). Transitions between the elongated tubules and the spindle cells are commonly seen, and in some tumors the spindle cell areas can be the dominant component, at times resembling a mesenchymal neoplasm such as leiomyoma or myofibroblastoma [13] (Fig. 2b). Papillation projections with tumor cell tufts protruding into the tubular lumen, and true papilla with well-shaped fibrovascular cores can be seen as a minor component [14, 13, 15–17, 6, 18], and rarely, as a prominent component [19] in MTSRCC. Extracellular blue-gray mucinous/myxoid matrix are usually abundant in the majority cases of MTSRCC, sometimes these mucinous collections may appear as numerous small vacuoles partially obscuring the MTSRCC architecture and mimicking clear cells [13] (Fig. 2c). A so-called “mucin-poor” pattern of MTSRCC has recently been described where there is little or no extracellular mucin that can be appreciable on routine microscopy (Fig. 2d), in this setting, Alcian blue stain can highlights the scant mucin in the tumor [13, 20]. Cytologically, the tumor cells are usually bland-appearing with scant, pale to slightly eosinophilic cytoplasm and indistinctive borders. Rarely, minor areas with clear cell and oncocytic changes have been reported [13, 17, 21] (Fig. 3a). The nuclei are generally round, uniform and display low nuclear grade characteristics with evenly dispersed chromatin and inconspicuous nucleoli corresponding to Fuhrman nuclear grade 2, but occasionally high nuclear grade change may be observed [22–25] (Fig. 3b). Mitoses are rare and necrosis is uncommonly seen. Examples of MTSRCC with sarcomatoid differentiation characterized by high-grade spindle cell proliferation with marked cytologic atypia, tumor necrosis, and increased mitotic activity have been recently reported [26–29] (Fig. 3c). In additional to myxoid degeneration, other common and not-so-common stromal changes that can be seen in MTSRCC include aggregations of foamy macrophages (Fig. 3d), cuffing infiltrations of lymphoplasmacytic cells surrounding the tumor cell nests (Fig. 3e), depositions of small psammoma bodies (Fig. 3f), and heterotopic bone formation.

**Fig. 2:** Microscopic features of MTSRCC. **a** The tumor is composed of elongated tubules and spindle cells that are separated by abundant basophilic extracellular mucinous stroma. **b** When spindle cells dominate, this tumor may mimics a mesenchymal tumor. **c** Occasionally, mucinous collections may appear as numerous small vacuoles (*arrow*) imparting an appearance of clear cells. **d** Depicting a mucin-poor pattern of MTSRCC

**Fig. 3:** Uncommon histologic features of MTSRCC. **a** Foci of clear cell changes. **b** High grade MTSRCC with prominent nucleoli corresponding to Fuhrman grade 3. **c** MTSRCC with sarcomatoid transformation (*left*, sarcomatoid component; *right*, mucin-poor MTSRCC). **d** Aggregations of foamy macrophages (*arrow*). **e** Cuffing infiltrations of lymphoplasmacytic cells. **f** Depositions of small psammoma bodies (*arrow*)

### Immunohistochemical findings

Immunohistochemical studies of MTSRCC show that the neoplastic cells of both the tubules and spindle cells stain consistently positively for PAX2/8, low molecular weight cytokeratins (CK8/18, CK19 and CK7) (Fig. 4a), epithelial membrane antigen (EMA), alpha-methylacyl-CoA racemase (AMACR) (Fig. 4b), and E-cadherin [30, 14, 15]. Staining for vimentin (Fig. 4c) and high molecular weight cytokeratin (34BE12) show variable expression, and RCC maker, CD10 and CD15 are often negative but occasionally be positive [15, 16], while staining for carbonic anhydrase IX, ulex europaeus agglutinin (UEA-1), P63, CK20, GATA3 and smooth muscle actin (SMA) are typically negative [30] (Table 1). Recently evidence of MTSRCC with neuroendocrine differentation, with tumor cells immunostaining for chromogranin A (Fig. 4d), synaptophysin, and neuron-specific enolase, have been reported, and in some cases supported by ultrastructural findings [31–33].

**Fig. 4:** Immunohistochemical features of MTSRCC. The neoplastic cells of both the tubules and spindle cells stain consistently positively for (**a**) CK7 and (**b**) AMACR. Most cases stain positively for (**c**) vimentin. A minority of cases may show neuroendocrine differentiation, as depicted here, express (**d**) chromogranin A

**Table 1:** Summary of immunohistochemical staining profile of MTSRCC

Authors (yr)	No. cases	AMACR	AE1/AE3	CK7	CK19	EMA	Vimentin	RCC maker	CD10	CD15	HMWCK	E-cadherin
Parwani et al. (2001) [3]	4	NA	4/4	4/4	0/4	4/4	4/4	NA	NA	0/4	4/4	NA
Rakozy et al. (2002) [4]	5	NA	5/5	NA	4/5	5/5	2/5	0/5	NA	NA	NA	NA
Hes et al. (2002) [5]	11	NA	11/11	9/9	NA	11/11	11/11	NA	NA	0/11	NA	NA
Ferlicot et al. (2005) [14]	15	12/12	13/13	14/14	13/13	14/14	2/14	5/11	3/14	4/14	3/14	10/11
Paner et al. (2006) [15]	27	25/27	NA	22/27	NA	19/20	NA	2/27	4/27	NA	4/26	NA
Fine et al. (2006) [13]	17	9/13	NA	12/13	NA	NA	NA	NP	NA	NA	NA	NA
Shen et al. (2007) [16]	12	11/12	NA	11/12	NA	NA	NA	11/12	6/12	11/12	NA	NA
Wu et al. (2014) [6]	8	7/8	NA	5/8	NA	3/8	6/8	NA	NA	NA	NA	NA

*HMWCK* high molecular weight CK, *NA* not available

### Histogenesis and molecular genetics

The ontogenic identity of epithelial nature between the tubular and spindle cell component in MTSRCC has been well established by immunohistochemisty, however, the exact renal epithelial cell line of differentiation remains debatable [15]. Although MTSRCC was initially considered to originate from either cells of the loop of Henle or collecting duct epithelium [2, 3, 34], accumulated evidence showing complex immunoprofile with uniform expression of CK7 and AMACR suggests its proximal nephron origin and intimate relationship to papillary RCC [15, 16, 7]. Indeed, some authors have suggested that MTSRCC may represents a variant of papillary RCC [16, 18], and in some settings, make a confident distinction between these two entities based on routine microscopy and immunohistochemistry may be impossible and often requires molecular genetic studies [8].

Genomic investigations for MTSRCC, mainly in single case or small series studies and based on karyotyping, comparative genomic hybridization (CGH), and fluorescent in situ hybridization (FISH) analyses, have demonstrated multiple chromosomal numerical aberrations in these tumors, with losses of (or partly from) chromosomes 1, 4, 6, 8, 9, 11, 13, 14, 15, 18, 22 and X, as well as gains of all or parts of chromosomes 2, 3, 4, 5, 7, 9, 10, 12, 15, 16, 17, 18, 19, 20, 22 and Y [3, 4, 14, 35, 28, 24] (Table 2). Most recently, Peckova et al. [25] who investigated hitherto the largest series of MTSRCC for molecular genetic abnormalities using CGH analysis found that both the low grade and high grade MTSRCC of classic morphology showed chromosomal losses including 1, 4, 6, 8, 9, 13, 14, 15, and 22 without any chromosomal ganis detected, while those showing morphologic features overlapping with papillary RCC demonstrated a more variable pattern with multiple chromosomal losses and gains, including gains of chromosomes 7 and 17 in two of the four analyzable tumors. However, FISH-based analyses have consistently proved that MTSRCC lacks of the the gains of chromosomes 7 and 17 and losses of chromosome Y that are characteristic of papillary RCC [36, 19]. These emerging evidence suggests that MTSRCC is histologically heterogenous tumor that can shows morphologic and immunohistochemical features overlapping with papillary RCC, but genetically distinctive entity different from papillary RCC.

**Table 2:** Summary of chromosomal aberrations of MTSRCC evaluated by CGH studies

Authors (yr)	No. cases	Histology	Chromosome losses	Chromosome gains
Rakozy et al. (2002) [4]	5	Classic MTSRCC	1, 4, 6, 8, 9, 13,14, 15, 22, X	
Ferlicot et al. (2005) [14]	2	Classic MTSRCC	1, 4, 6, 8, 11, 13, 14, 15, 18, 22	15
Brandal et al. (2006) [35]	2	Classic MTSRCC	1, 6, 8, 9, 10, 11, 13, 14, 15, 22	2, 4, 7, 16, 17, 18, 20
Dhillon et al. (2009) [28]	1	Sarcomatoid MTSRCC	14, 15	2, 5, 7, 9, 10, 12, 17, 19, 20, 22, X
Kuroda et al. (2011) [24]	1	High-grade MTSRCC	1, 6, 8, 11, 13	1, 7, 16, 19, Y
Peckova et al. (2015) [25]	4	Classic MTSRCC	1, 4, 8, 9, 14, 15, 22	
	4	High-grade MTSRCC	1, 4, 6, 8, 9, 13, 14, 15, 22	
	4	MTSRCC overlapping with papillary RCC	1, 6, 8, 9, 14, 15, 22	3, 7, 16, 17

### Differential diagnosis

MTSRCC in its classic form is so distinctive that there should be no diagnostic problem, however, when variant patterns of the tumor are seen, such as predominance of spindle cells, paucity of mucin, diagnostic difficulties may arise, particularly on needle biopsies when pathologists are providing with only tiny materials. With regard to MTSRCC where spindle cells dominate, the most critical differential diagnosis is sarcomatoid RCC, which can develops in any form of RCC and usually confers an aggressive behavior. The spindle cells in MTSRCC are bland-looking with uniform architectural pattern and usually low nuclear grade, lacking large, hyperchromatic/pleomorphic nuclei, significant mitotic activity or sheet of necrosis which are prevalent in sarcomatoid RCC. MTSRCC itself can experiences sarcomatoid transformation [28], however, in these tumors, at least focally, evidence of a low grade component exists. Spindle cell predominant MTSRCC may be confused with mesenchymal neoplasms such as smooth muscle tumors (both leiomyoma and leiomyosarcoma), and inflammatory myofibroblastic tumor (IMT) when infiltrated by severe chronic inflammations. However, both smooth muscle tumors and IMT usually have a more distinct fascicular arrangement and more elongated nuclei, and label strongly with SMA and rarely with cytokeratins. Lastly, as above have mentioned, overlapping morphologic features with papillary RCC can make the distinction between MTSRCC and papillary RCC difficult. Type 1 papillary RCC in areas can adopts a solid growth pattern with compression of elongated tubules and papillae which imparts a fusiform architecture mimicing MTSRCC. However, papillary RCC usually has a predominantly tubulopapillary pattern with complex branching papilla containing well-deformed fibrovascular cores and lacks of mucinous stroma which usually extensively and at least focally exist in MTSRCC. Immunocytochemistry in distinguishing papillary RCC from MTSRCC is largely unhelpful because the two entities share a CK7 and AMACR positive profile, although CD10 is less likely to be reactive in MTSRCC than in papillary RCC [15]. Recently, a so-called papillary RCC with low grade spindle cell foci has been described which can shows morphology significantly resembling MTSRCC [37]. In contrast to MTSRCC, this tumor is characterized by a male predominance and foci of bland-appearing spindle cells dispersed among more conventional looking papillary RCC. As this tumor dispalys the typical gains of chromosomes 7 and 17 associated with papillary RCC, FISH analysis can be used to clinch the diagnosis if needed [37].

### Prognosis and therapy

The prognosis for MTSRCC with classic morphology is generally favorable and complete surgical excision appears to be adequate treatment [1]. These tumors are generally of low pathological stage (pT1, pT2) at diagnosis and are amenable to partial or radical nephrectomy. Few cases have demonstrated tumor recurrence, regional lymph nodes and distant sites metastases, as well as tumor-associated deaths [3, 5, 4, 14, 26, 28, 38, 39]. Metastasis usually occurs in tumors with atypical histological features such as high nuclear grade and sarcomatoid transformation, however, cases with classic, low-grade morphology of MTSRCC developing multiple distant metastases with both the primary tumor and metastases displaying identical morphology have also been reported [38, 39]. It is therefore recommended that although an innocent outcome is likely, a close follow-up is warranted. With regard to the therapy of MTSRCC, patients with localised disease are usually treated with resection, either partial or radical nephrectomy. For metastatic diseases, there are no reports of systemic treatment guideline published to date. Most recently one case of metastatic MTSRCC showing a response to sunitinib has been documented [40].

## Conclusions

Although a close relationship to papillary RCC has been suggested, on the basis of clinical, morphological as well as molecular genetic data, we consider MTSRCC to be a separate and distinct renal neoplastic entity. This tumor has a histological spectrum ranging from low to high grade that includes sarcomatoid differentiation which can confers the tumor an aggressive clinical course.
